# Implementation of Short Video Click-Through Rate Estimation Model Based on Cross-Media Collaborative Filtering Neural Network

**DOI:** 10.1155/2022/4951912

**Published:** 2022-05-31

**Authors:** Ying Feng, Guisheng Zhao

**Affiliations:** ^1^Shandong Women's University, Shandong, Jinan 250300, China; ^2^School of Film and Television Media, Shanghai Normal University, Shanghai 200234, China

## Abstract

In this paper, we analyze the construction of cross-media collaborative filtering neural network model to design an in-depth model for fast video click-through rate projection based on cross-media collaborative filtering neural network. In this paper, by directly extracting the image features, behavioral features, and audio features of short videos as video feature representation, more video information is considered than other models. The experimental results show that the model incorporating multimodal elements improves AUC performance metrics compared to those without multimodal features. In this paper, we take advantage of recurrent neural networks in processing sequence information and incorporate them into the deep-width model to make up for the lack of capability of the original deep-width model in learning the dependencies between user sequence data and propose a deep-width model based on attention mechanism to model users' historical behaviors and explore the influence of different historical behaviors of users on current behaviors using the attention mechanism. Data augmentation techniques are used to deal with cases where the length of user behavior sequences is too short. This paper uses the input layer and top connection when introducing historical behavior sequences. The models commonly used in recent years are selected for comparison, and the experimental results show that the proposed model improves in AUC, accuracy, and log loss metrics.

## 1. Introduction

In recent years, deep learning has achieved great success in computer vision. Deep convolutional neural networks, built to mimic the neural mechanisms of the human visual cortex, can mine the underlying features of images and are widely used in image classification and recognition [1]. Deep learning algorithms are computational and storage-intensive, and deep convolutional neural networks enhance their expressive power by increasing depth, trading time, and space for higher-level abstract features [2]. Researchers use deep compression to significantly reduce the computational and and storage requirements required by neural networks to address this limitation. In the face of massive multimedia data, deep learning for cross-media retrieval has become a hot research topic today. In this paper, deep learning methods are used in cross-media retrieval to make full use of its abstraction ability to learn correlations between different modal media and to address the problems of computationally intensive and slow deep neural network models; we propose a cross-media retrieval method based on compressed convolutional neural networks to improve retrieval speed while ensuring retrieval accuracy.

Nowadays, recommendation systems are used in e-commerce platforms, blogs, movie sites, personalized music software, social networking sites, etc. Each area and venue has its recommendation characteristics [3]. With the rapid development of the network economy, the recommendation system plays an increasingly important role. The logistic regression model mainly relies on the manual construction of valuable features, and then after the linear transformation of the features, the values are mapped between [0, 1] by the sigmoid function as the predicted values of the click-through rate. The memory-based collaborative filtering recommendation algorithm is also called a neighborhood-based recommendation. The memory-based collaborative filtering recommendation algorithm is divided into User-based Collaborative Filtering and Project-based Collaborative Filtering. Model-based Collaborative Filtering recommendation algorithms can be divided into matrix decomposition-based, clustering-based, etc. [4]. The basic principle can be understood by converting the user-project scoring matrix into different models and then using these models in different application scenarios to recommend items to users.

The vast amount of user-generated content, video uploads, and updates makes the number of resources in the network grow exponentially, which brings the problem of “information overload” and “information explosion.” Collaborative filtering techniques can be classified into Memory-based CF and Model-based CF based on whether they are modeled using machine learning ideas. The matrix decomposition method of model-based collaborative filtering is popular because it is easy to implement and expand in multiple perspectives in neural networks. It is challenging to dig out valuable information for users and platforms from the vast amount of short video data and help temporary video platforms distribute and attract traffic, directly affecting the platform's revenue and users' experience [5]. Click-through rate prediction is an integral part of this task, and how to improve the accuracy of click-through rate prediction for short videos has attracted extensive attention from academia and the industry [6]. The Click-Through Rate (CTR) problem predicts the probability that a user will click on an item given a context. In the field of recommendation, since the expected click-through rate reflects the user's interest in an item, the predicted click-through rate can be ranked to form a proper recommendation sequence to achieve a thousand people's personalized recommendation effect. With the gradual development of computer vision and natural language processing, the problem of predicting click-through rate by integrating visual and textual information has become one of the famous research directions.

## 2. Related Works

The standard recommendation algorithms include the user-based collaborative filtering algorithm, and item-based and content-based recommendation algorithm. The user-based collaborative filtering algorithm has the most extended history, and the item-based collaborative filtering algorithm is the most widely used. The collaborative filtering algorithm is a neighborhood algorithm [7]. The main idea is to calculate the degree of similarity of users or items by calculating the cosine similarity of users or objects. Collaborative filtering techniques can be classified as Memory-based CF and Model-based CF according to whether they are modeled using machine learning ideas. Among the model-based collaborative filtering methods, matrix decomposition is popular because it is easy to implement and expand in multiple neural network perspectives [8]. The mathematical singular value decomposition method SVD decomposition takes the form of multiplying three matrices. The left and right matrices represent user and item implied factor matrices, respectively, and the middle matrix is a singular value matrix and is a diagonal matrix. Each element satisfies each element's nonnegativity and decreases gradually [9]. We can call this mathematical matrix decomposition method as Pure SVD, which has an essential requirement for the original matrix—the original matrix is dense, i.e., there are no nonempty elements in the original matrix, and at the same time, the time complexity of Pure SVD is *O*(*n*^3^), which is not suitable for large data operations. Later, Ge et al. proposed the Funk SVD method, which no longer decomposes the matrix into three matrices but reduces the computational complexity by decomposing the matrix into two matrices and letting the new matrix obtained by matrix multiplication of these two matrices have a reduced error with the original matrix [10]. Funk SVD has practical physical significance in recommender systems and promotes the development of hidden semantic models in recommender systems.

The Click-through rate is one of the core bases for Internet companies to allocate traffic. For example, for Internet advertising platforms, accurate click-through rate prediction is indispensable to finely weigh and protect users' interests, advertisers, and media. Click-through rate prediction techniques range from traditional logistic regression (LR) to deep learning, which has been a big hit in the past two years, and new algorithms have emerged, such as Deep FM, DIN, etc. In this paper, click-through rate prediction models are classified into three major categories from feature utilization, namely, shallow models, deep models, and hybrid models [11]. The most classic of the external models is the logistic regression model, which has the features of simple logic, easy parallelization implementation, and strong interpretability, so it is often used as the baseline model in the industry. The logistic regression model mainly relies on the manual construction of practical features. Then, after the linear transformation of the features, the value is mapped to between [0, 1] by the sigmoid function as the prediction value of the click rate [12]. Logistic regression models are more suitable for modeling dense data, but in the scenario of click-through rate prediction, the information is often very dimensional and sparse. Therefore, Hew and Lo proposed a hash method to map high-dimensional light features to low-dimensional dense features, which proved simple and effective [13]. Elbalka et al. presented the FTRL (Follow the Regularized Leader) algorithm, which made a lot of engineering optimizations to the logistic regression model, making it more suitable for practical applications online [14]. It was more convenient for online use in practical applications. However, it is still essentially a linear model, which cannot handle the nonlinear relationship between features and targets, so the model effect depends heavily on the feature engineering experience of algorithm engineers.

In 1992, Tang and other scholars first proposed a recommendation system and successfully applied the technology to the Tapestry e-mail system [15]. The Group Lens Research group at the University of Minnesota then improved the personalized recommendation algorithm by developing an automated collaborative filtering algorithm that can automatically find the set of neighboring users of a target user in the system, which was also successfully applied to the Movie Lens movie recommendation system developed by the group [16]. In the study of a user-based collaborative filtering algorithm, Han et al. proposed an improved user-based improved collaborative filtering algorithm by combining rated item pooling (RIP) with a more detailed comparison of user attributes in RIP to improve the similarity calculation method [17]. Dividing items into different RIPs based on other preferences of users provides a basis for fine-grained calculation of similarity between users, which can help the model build the set of near-neighboring users more accurately and thus improve recommendation accuracy. Hu et al. classified users into three categories, namely, exceptionally similar, average similar, and very dissimilar, based on the traditional similarity calculation method between users [18]. Tong et al. proposed an improved similarity calculation method for the average similar users [19]. The experimental results showed that the process could further reduce the error and improve the hit rate of recommendation. The results show that the method has high recommendation accuracy in the cold start case.

## 3. Design of Short Video Click-Through Rate Imputation Model Based on Cross-Media Collaborative Filtering Neural Network

### 3.1. Cross-Media Model Construction

Science and technology big data contain a large amount of relevant data; there is a lot of noise and very little practical information. Therefore, how to filter out the noise information widely existing in the science and technology big data in a wide range of data, obtain the attribute data related to the science and technology big data object itself and the published content message, and doing a good job in data preprocessing and storage according to the category is very important for the follow-up research. The flow chart of data collection, processing, and storage is shown in Figure 1. The existing crawler system is used to crawl the data according to the four aspects of keywords, time range, crawl depth, and essential attributes of cross-media technology big data as the input parameters of the crawler, so that the corresponding categorized data can be obtained according to the name of cross-media technology big data. At the same time, for the crawled data, such as policy text data, extract the time, region, department, and other attributes issued by the policy text and process it for subsequent research. This way, we can obtain the processed cross-media science and technology extensive data text dataset, storing information such as policy text, policy title, policy link, release time, release unit, keywords, and support type. Researchers have used deep compression to significantly reduce neural networks' computational and storage requirements to address this limitation. In the face of massive amounts of multimedia data, deep learning for cross-media retrieval has become a hot research topic today.

Determine the subject keywords of the policy data of cross-media science and big technology data, and then the search port of the official website of information disclosure for the collection of policy data of science and technology big data, and collect the data of the corresponding publishing regions, policy links, policy titles, policy keywords, etc., while collecting the original text information. Due to the data structure characteristics of the ordered data sets, different data acquisition methods are required for different types of data structures. The distributed crawler framework is used to complete the data crawling. The steps of the crawler are mainly divided into the following steps: first, browse the website content to select the list of links to build the websites to be crawled, then traverse each list of websites in turn, and for the structured data websites, crawl directly according to the tags, for the unstructured data websites, we select the crawled content based on keyword search, and shuffle the formatted data that are now stored according to the original format, and the crawled unstructured data are separately distinguished from carrying out the subsequent data processing operations.

For the text data of science and technology, the original text data are corpus cleaned, and the text content is uniformly formatted and denoised. Based on the regular expression matching rules, text data matching with features in text can be extracted [20]. In this way, the text dataset under the processed science and technology big data can be obtained. In addition, since the dataset crawled in this paper is mainly unstructured data, most of them are an article or a phrase, etc., which cannot be used directly [21]. Therefore, after crawling the raw unstructured data, we need to perform word separation and linguistic analysis on the crawled raw unstructured data. After word separation, valuable knowledge is selected based on linguistic properties, and useless modifier words are discarded. After processing the raw data based on word separation and deactivation, each word group afterword separation is converted into a model vector by the worded model, thus mapping the text data of big data into its corresponding matrix-vector, and a word vector can be used for big data of science and technology.

### 3.2. Collaborative Filtering Neural Network Model Design

Traditional user-based approaches calculate the similarity values between users using their interaction data vectors with a specific similarity calculation function and weight the items with scores based on the similarity between users. Such an approach relies heavily on the data density of the scoring matrix. Still, realistic data are often very sparse, and users may rarely share preferred items, which significantly impact the recommendation effectiveness of this approach. The basic structure of a convolutional neural network collaborative filtering model based on the outer vector product is given, as shown in Figure 2. The model's input consists of an interaction graph obtained by the exterior product of the user vector and the item vector. In the neural network layer part of this paper, the convolutional neural network, which is the best at processing graphs, is chosen. Model-based collaborative filtering recommendation algorithms can be divided into matrix decomposition-based, clustering-based, etc. The basic principle can be understood by transforming the user-item rating matrix into different models and then using these models in different application scenarios to recommend items to users. The prediction layer will make the final user preference prediction based on the features extracted from the convolutional layer. A typical example of this model is the Conv NCF, whose convolutional layer uses a complete convolutional neural network with a convolutional kernel size of 2 × 2 and a step size of 2 until the final feature map (the topmost feature map) is mapped to a value. Then, the vector composed of all the convolutional feature maps (discounts, at which point only one value remains in the feature map) is fed into the prediction layer. The convolutional layer here can be applied to a variety of convolutional neural network structures without being limited to a specific form; however, both in theory and in practical application results, the depth of the convolutional network has a particular influence on the performance of the model, i.e., it should not be too deep.

From a theoretical analysis, we know that convolutional networks are used for local feature extraction on the one hand and focus on specific valuable parts of local features on the other hand, which are then passed to the upper layers of the network. This means that each layer of the convolutional network deliberately “filters out” some of the information to leave the most valuable part for prediction. The reason for performing dimensionality reduction is that processing and analyzing high-dimensional features require a lot of computational resources and even generate dimensional disasters, so it is essential to represent the original high-dimensional feature vector with a low-dimensional feature vector. However, as analyzed in the previous section, the entire prediction model requires backpropagation of the target loss to train the user and item vectors, i.e., the values of the feature maps are derived from the loss gradient of the target function [22]. This makes the training results of the model, i.e., the final user vector and item vector contain more information from the training set, which means they are easy to be overfitted. From the actual experimental results, we find that not only the depth of the convolutional network here degrades the performance of the model but also the multi-layer perceptron co-filtering model based on the splicing vectors and the co-filtering model based on the stacked vectors of the convolutional neural network proposed in this paper have similar findings. The Steck NCF model is mainly divided into a track composed of implicit factors, an association relationship processing model between implicit factor dimensions (only convolutional network models are considered in SECk NCF), and a target prediction mapping layer. The model is divided into a tracklayer, a hidden layer, and a prediction layer.

(1) Crawler layer: In simple collaborative filtering, we will only use the index of the user and the index of the item as the only input information to the model, and in the two SECk NCF examples we give, we also use only the indexes of the user and the item. Thus, we can obtain the vector *P*_*u*_ ∈ *R*^*k*^ for user *u* and thing *i*, where *K* is the dimensionality of the vector. Take *D*_*u*_^*K*×*K*^ ∈ *R*^*K*×*K*^ to denote the track's words *K* × *K*, where *u* denotes any user *u* and *i* denotes an item *i*.
  (1) $$\begin{array}{c} D_{u}^{K}=\sum S\left(P_{u}-Q_{i}\right),\\ D_{ui}^{K}=\sum_{i=1}\frac{P_{u}-Q_{i}}{\sqrt{P-Q}}. \end{array}$$
(2) Hidden layers: A set of hidden layers is used to extract valuable implicit factor dimensional correlation signals on top of the crawler layer. Here, a complex design can be used to obtain more valuable indications. If the parameters of the hidden layers are denoted by *θ*, the formula for the output vector of the hidden layers can be obtained: Content-based collaborative filtering algorithms are popular in personalization applications. The similarity is calculated based on the popularity of two items or content, and similar items or content are recommended for users to explore their potential associations, being insensitive to the addition of new content and allowing the data to be expanded at will.
  (2) $$\begin{array}{c} v_{\left(\text{hidden}\right)}=\int_{\theta }\frac{D^{K}}{\sqrt{D^{ui}-1}}. \end{array}$$
Here *fθ* denotes the hidden layer model with *θ* as a parameter, and *v*hidden represents the final output of the remote layer vector provided to the prediction layer for predicting the outcome. It is worth noting that the hidden layer model here needs to be specially designed to accept the crawler layer as input to capture valuable and valuable signals of correlation information between dimensions.
(3) Prediction layer: The prediction layer accepts the vector *v*hidden from the output of the hidden layer. These vectors successfully capture the various possible interaction associations between dimensions, and we can calculate the estimation result by using the equation. Here *w* denotes the weight of each element of the parameter representation vector *v*hidden in the prediction layer. In contrast, aout indicates the activation function of the output layer, and for implicit feedback, aout is usually a sigmoid function, i.e., (*x*) = 1/(1 + *e* − *x*). Finally, to conclude, the parameters of the whole SECk NCF model are: *θ*, *P*, *Q*, *w*
  (3) $$\begin{array}{c} y_{u-i}=\sum \text{out}\left(w^{t+1}-v_{\text{hidden}}\right). \end{array}$$
(4) SECk NCF prediction model learning: According to the pointwise loss method based on single-category prediction proposed in the NCF article, taking 1 indicates the presence of user-item interaction and 0 the other way around. Therefore, we need to limit the final output prediction value *y*^*u*, *i* to 5 between [0, 1], which is, of course, easily achieved by a probabilistic function, such as a logistic function as the activation function of the prediction layer. Based on the above parameter settings, the likelihood function is given here: The image feature is essential in video content analysis, often used in target detection, scene recognition, and other fields. It is derived by segmenting the video into frames and extracted by CNN for video frames.
  (4) $$\begin{array}{c} P_{\left(\theta ,P,Q,w\right)}=\frac{\sum \left(u+i\right)}{\sum_{u=1}\left(1-y_{u-i}\right)}. \end{array}$$
(5) Motivation for using convolutional neural networks
The hidden layer can also use MLP (by flattening the tracklayer). Still, it loses the dimensional pairwise and locally tightly connected nature of the track. Note that after Flat, the tracklayer is transformed into a *k* ∗ *K* dimensional vector, consistent with the approach in NCF. However, MLP is theoretically able to fit arbitrary approximation functions. This requires a large amount of experimental data to drive the results; however, real-life data are primarily sparse and leads to suboptimal outcomes. On the other hand, using MLP often requires a larger vector dimension *K* and a deeper network hierarchy, but this also leads to problems such as the parameters of the network becoming inaccessible, large, and complex for real machines to process at high speed. These problems can be solved very well using convolutional networks. Conversely, convolutional networks are very good at handling local feature relationships. The number of feature maps or kernels can determine how many correlations exist between regional dimensions, thus generating wealthy inter-dimensional interaction information. On the other hand, existing neural network frameworks can use the parallel computing power of CPUs or GPUs for convolutional networks to achieve high-speed processing, making such models realistic and feasible.

### 3.3. Short Video Click-Through Rate Projection Model Design

Image feature is the essential feature in video content analysis, which is often used in target detection, scene recognition, and other fields. It is derived by segmenting the video into frames and extracted by CNN for video frames. The most used in previous research work are VGGNet and Alex Net implementations. These models have a low number of network layers and a low computational complexity. However, ZDNet visualizes the intermediate hidden convolutional layers and finds that the more profound the CNN network layers are, the richer the extracted image features are, and the more semantic information can be expressed. However, there is also a network degradation problem when the number of network layers increases. Therefore, this paper chooses the residual neural network Res Net152 to extract image features because it incorporates the residual module to ensure that the model will not degrade with deeper depth. In this paper, before using the ResNet152 model for feature extraction, we use the Image Net dataset for pretraining of classification, which helps the model recognize many object types in short videos. In the experiments, this paper chooses the output of the last fully connected layer as the feature representation of RGB images with 1000 dimensions. The behavioral feature, also known as the Spatio-Temporal Feature, is often used in areas such as video behavior recognition, which is extracted using a 3D convolutional network. The Click-Through Rate (CTR) problem predicts the probability of a user clicking on an item given a context. Since the expected click-through rate reflects the user's interest in an item, the expected click-through rate can be ranked to form a proper recommendation sequence, thus realizing the personalized recommendation effect of a thousand people. Since it can model both spatial and temporal dimensions, this feature is introduced in this paper for learning the behaviors contained in the videos. Since the number of video frames in the dataset is inconsistent, this paper first obtains a fixed-length vector as a feature representation of the video by sequentially sampling *N* frames from the video and then using the *N* frames as the input to the 3D convolutional network. This paper uses the C3D network for extraction after pretraining on the Sport-1M dataset, which helps the model identify the behavioral categories in short videos. In the experiments, this paper selected the output of the penultimate fully connected layer as the behavioral video features with 4096 dimensions. The audio in the video also contains rich information, even information that cannot be captured visually, such as the surrounding environment and emotion. Mel Frequency Cepstral Coefficients (MFCC) is a typical representation of audio features obtained by first converting the audio signal to Mel frequency and then performing cepstral analysis [23]. In addition, there are other standard features, such as spectral spread, energy entropy, and over-zero rate, and the details are shown in Table 1. There are many mature methods for extracting audio features, and an open-source pie Audio Analysis tool is used in this paper. In this paper, we first use the tool MPEG to remove the audio file from the video and then use the tool to extract the 34-dimensional features.

After obtaining each modal feature of the short video by the above independent feature extraction model, it needs to be fused to input the click-through rate prediction model. The image and behavioral features are first dimensionalized and normalized, and finally, all parts are naturally stitched to obtain a fixed-length feature vector. Performing dimensionality reduction is that processing and analyzing high-dimensional features requires a lot of computational resources and even generates dimensional disasters, so it is essential to represent the original high-dimensional feature vector with a low-dimensional feature vector. The dimensionality reduction method used in this article is principal component analysis, which is based on the principle of converting the original data represented by linearly correlated variables into a few data represented by linearly uncorrelated variables using orthogonal transformations, which are called principal components and may make the data with the most significant variance in the direction of principal components. Thus, it can reduce the feature dimensionality while retaining most of the information in the original data. The dimensionality of image features is reduced to 80 dimensions while having 99% of the information, and the dimensionality of behavioral features is reduced to 160 dimensions after dimensionality reduction. The reason for data normalization is that the dimensionality of each modal feature is different, so to eliminate the influence of the dimensionality between elements and make each modal part comparable, data normalization is required. The joint data normalization operations are max-min normalization and z-score normalization. Max-min normalization is a linear transformation of the original data so that the result falls between [0, 1]. Z-score normalization is a linear transformation of the original data so that the result falls between [0, 1]. Z-score normalization transforms the actual data distribution into a data distribution with mean 0 and variance 1. Analyzed from the perspective of gradient descent, the normalized data can find the optimal solution more easily with the same learning rate. The logistic regression model mainly relies on the manual construction of valuable features, and then after the linear transformation of the features, the values are mapped between [0, 1] by the sigmoid function as the predicted values of the click-through rate.

(5) $$\begin{array}{c} x_{\max-1}=\frac{x_{\max}+x_{\min}}{\sqrt{x_{\min}-1}}. \end{array}$$

The overall structure of the click-through rate prediction model is designed, which is obtained by combining GRU improvements with the DIN model. The model consists of a three-layer network structure. The first layer is the Embedding Layer, which is used for data preprocessing; the second layer is the Interest Evolution Layer, which is used for mining the interest behind the user's historical behavior and learning its evolution process; the third layer is the CTR Prediction Layer, which is used for understanding the third layer is the CTR Prediction Layer, which is used to learn higher-order combinations of features and obtain click-through rate prediction values. The interest evolution layer is the key to processing user behavior data and is the innovation of the MMIE model. The network structure of the click-through rate prediction model is shown in Figure 3. We know that convolutional networks are used to extract local features on the one hand and focus on specific valuable parts of the local features on the other hand, which are then passed to the upper layers of the network. This means that each layer of the convolutional network deliberately “filters out” some of the information to leave the most valuable part of the information for prediction.

The model's input includes user behavior sequence, target video, and other features (including contextual features, user ID, etc.). Suppose the elements of the user behavior sequence are represented as *x* = [*v*_1_, *v*_2_ … *v*_*h*_]^*T*^, where *v*_*i*_ represents the feature vector of the *i*th behavior of the video in the user behavior sequence, *H* represents the length of the user behavior sequence, *v*_*i*_ = [*v*_*ir*_, *v*_*ic*_, *v*_*iA*_]^*T*^ means the *i*th video contains image features, behavior features, and audio features; the features of the target video are *v*_*a*_ = [*v*_*ar*_, *v*_*ac*_, *v*_*aA*_]^*T*^, and other features are represented as *v*_*c*_. The embedding layer needs to learn the mapping matrix *W*_*j*_ = [*w*_*j*1_, *w*_*j*2_…*w*_*jk*_] ∈ *R*^*D*×*K*^, which means the mapping matrix of class *j* elements, *D* represents the dimensionality of the original features, and *K*_*j*_ represents the dimensionality of the mapped features. Then, after the embedding layer*e*_*c*_, the original behavioral sequence features are noted as*e* = [*e*_*i*1_, *e*_*i*2_,…*e*_*iH*_]^*T*^ = [*w*_*i*1_, *w*_*i*2_,…*w*_*iH*_], and the post-embedding features of other features are pointed out as *e*_*c*_. The user behavioral sequence needs to go through the interest evolution layer to mine the user interest representation behind it, and the formula can express its operation process: The recommendation system is not only applied to e-commerce platforms but also blogs, movie sites, personalized music software, social networking sites, and other platform sites all use the recommendation system to varying degrees, and each area and platform has its recommendation features.

(6) $$\begin{array}{c} \text{soft}\max\left(f-1\right)=\frac{\exp\left(\theta +f\right)}{\sqrt{\sum \exp\left(\theta_{k-1}-f\right)}}. \end{array}$$

## 4. Analysis of Results

### 4.1. Analysis of Cross-Media Collaborative Filtering Neural Network Model

After the construction of Transmedia Technology, Big Data Knowledge Graph de is completed; the original lengthy text data can be vividly visualized with the help of knowledge graph technology. Based on the proposed BERT-BLSTM-CRF-based entity identification algorithm and BGRU-ATTENTION-based entity relationship extraction algorithm, the time series dimension is introduced to extend our database by automatically acquiring the latest data daily to achieve the dynamic portrait of science and technology resources [24]. The most mainstream Bayesian method in traditional machine learning is introduced to improve the accuracy of the vibrant picture of science and technology resources and solve the problem that the photograph's accuracy is affected by the multiple meanings the data expansion brings. The newly acquired science and technology data and the data in the database are firstly disambiguated after the daily dynamic data acquisition to avoid the decrease in the accuracy of the portrait brought by the entity disambiguation. After determining the evaluation indexes for this experiment, the paper's author information has more information than other attributes such as title and abstract. The data features selected to extract the author attributes separately and other attributes of the paper were compared with the current mainstream classification models in traditional machine learning to carry out the experiments in turn. The experimental results of these models in separate feature extraction are shown in Figure 4.

Content-based collaborative filtering algorithm (Item CF) extracts the features to be concerned from the filtered objects, uses their features to calculate the similarity, and then uses the preferences of different users to generate a recommendation list. The content-based collaborative filtering algorithm is popular in personalization applications. It calculates similarity based on the popularity of two items or contents, recommends similar items or contents for users to explore their potential associations, is insensitive to the addition of new content, and expands the data at will. A typical example of the model is the Conv NCF, whose convolutional layer uses a complete convolutional neural network with a convolutional kernel size of 2 × 2 and a step size of 2 until the final feature map (the topmost feature map) is mapped to a value, and then the vector composed of all the convolutional feature maps (discounts, at which point only one value remains in the feature map) is fed into the prediction layer. The recommendation of a user-based collaborative filtering algorithm is based on the similarity between users to find the group of users like the target users. In this similar group of users, items unknown to the target users but generally liked are recommended to the target users. Calculating the inter-user similarity can be implemented using Jaccard's formula, where the user's interest in the item is used as a behavioral indicator to calculate the inter-user similarity. *K* users like the target user are formed into identical user groups based on the computer user similarity. The items of general interest from similar user groups are used to find the potential content of interest unknown to the target user.

(7) $$\begin{array}{c} w_{u-v}=\sum \frac{\sqrt{n\left(u\right)-n\left(v\right)}}{\sqrt{n\left(u\right)+n\left(v\right)}}. \end{array}$$

We use Kera's to implement our model. We randomly select a training sample from the training set as the validation set for super parameter conditioning and then make predictions on the test set. We sample 4 negative sample instances for each positive sample instance by default [25]. For a reasonable comparison, we set the embedding size of all models to 64, use a Gaussian distribution (mean of 0 and 0.01) to initialize the parameters of the models, and use Adam for pointwise optimization with 256 as the default batch size and 0.001 as the default learning rate. Adam is an alternative optimization algorithm to stochastic gradient descent (SGD). Unlike the traditional stochastic gradient descent optimization algorithm, which always maintains a single learning rate and does not change during the training process, Adam calculates first-order and second-order moments for the parameters. He thus designs different adaptive learning rates for other parameters. Adam combines the advantages of Ada Grad and RMSProp. The adaptive gradient algorithm (Ada Grad) retains a learning rate for each parameter to improve performance on sparse gradients. At the same time, the root means square propagation algorithm (Respro) adaptively controls a learning rate for each parameter based on the mean of the nearest order of magnitude of the weight gradient, giving the algorithm excellent performance on nonstationary problems. 100k dataset is shown in Figure 5.

For MLP and Neu MF, we use the same structural configuration as in the NCF article and verify the effect of different embedding sizes. Finally, we find that the best performance is achieved for MLP with embedding size 64 in all three datasets. In contrast, the best results are achieved for both the MLP and GMF sides of Neu MF with Embedding. The best results were obtained for both the MLP and GMF sides of Neu MF with an embedding size of 64. We also tested the Neu MF pretrained with MLP and found no significant change in performance, i.e., no significant improvement. We also used BPR for personalized ranking on these three datasets. Deep learning algorithms are compute-intensive and storage-intensive. Deep convolutional neural networks enhance their expressive power by increasing their depth, trading time, and space for more advanced abstract features. Still, we do not report the experimental results of the BPR algorithm because all three datasets are too sparse to make the BPR algorithm perform poorly. The social network's extensive data search system includes a social network cross-media information real-time collection module, national security event cross-media feature extraction and search module, and social network content and user feature analysis module. Social network cross-media information real-time collection module: collects cross-media data from microblogs, saves the collected raw data from documenting database, synchronizes it to Elasticsearch regularly, and builds index. National security event cross-media feature extraction and search module: feature extraction of social network cross-media information, the introduction of irrelevant information filtering function of social network national security event, and semantic expansion search function of social network cross-media in the social network national security search system.

### 4.2. Short Video Click-Through Rate Projection Model Simulation Test

The experiments in this paper are run on a Linux server with 4 graphics cards (GPUs); the GPU model is TeslaK20m. All models are implemented using python 3.5 and Tensorflow 1.4. The size of Embedding was set to 128 for all models; the batch size was set to 32, the learning rate was 0.1 and gradually decreased to 0.01. Sequence segments were segmented at 30-minute intervals, and each piece was restricted to contain the five most recent behaviors, while only the ten most recent subsequences were used. Behaviors that exceeded the limit were discarded, and vice versa were made up. The performance of the MMIE and SDIN models was investigated for different sequence lengths [26]. The comparative experimental results of MMIE and SDIN models on short video datasets with varying sequence sizes are shown in Figure 6. In this subsection, after the model is trained, the test is summarized for different lengths of user behavior sequence data, and the sequence lengths are divided into seven groups [≤10, 11–15, 16–20, 21–25, 29–30, 31–35, >35]. The MMIE model has limited ability to model long sequence data, while the experimental performance of the SDIN model is better than MMIE. However, the experimental results of the SDIN model slowed down the growth trend with sequence length, suggesting that in the short video domain, the influence of past behaviors on current user interest becomes smaller with time growth.

The SDIN model achieves the best experimental results from the comparative exploratory analysis with other models. The SDIN model is a combination of several components, so this subsection examines the contribution of each element of the SDIN model to the final experimental performance. This subsection analyzes the contribution of each aspect of the SDIN model using the structural exclusion method. The attention mechanism is removed from the SDIN model. The average pooling operation is used instead of the attention mechanism, i.e., the model cannot achieve the adaptive generation of user interest representation in the face of different target items; the skin-II model, i.e., the intra-segment interest feature is removed from the SDIN model *I*, i.e., *I* is only used for the learning of inter-segment interest table and not for the teaching of higher-order cross features; SDIN-SII model, i.e., inter-segment interest features are removed from the SDIN model *H*, i.e., the learning of inter-segment interest evolution process is missing. This subsection still uses the contribution degree to measure the effectiveness of each component. All components contribute positively to the SDIN model. The inter-segment interest feature has the highest contribution to the model with a gift of 1.42%, indicating a temporal relationship between segment interest differences. Learning the temporal relationship in user interest is the key to improving the model's prediction accuracy. The comparison test results of different components are shown in Figure 7.

SDIN and SDIN&FM models perform better than other models on both datasets, e.g., the SDIN model has a 1.28% higher AUC value than the MMIE model on the short video dataset. And comparing the models implemented based on the same sequential segmentation idea, the SDIN model has a 1.1% higher AUC value than the HRNN model. Since the SDIN model also adds an attention mechanism compared with HRNN, the SDIN model is still 0.88% higher in the Arnett model comparison, indicating that the self-attention tool is more vital than RNN in modeling sequential data. And comparing the SDIN&FM model with the SDIN model, it can be found that the SDIN&FM model performs 0.11% higher than SDIN; however, the improvement of the experimental results is not significant, but it still indicates that the lower-order crossover features contribute to the effect of the model. Perhaps, other ways of combining lower-order crossover features should be used.

## 5. Conclusion

The rise of short video platforms has enriched people's entertainment life. Still, the ensuing massive number of short videos hinders users from accurately accessing the video content they are interested in. As an essential part of solving this problem, click-through rate estimation has received much attention from relevant research institutions and major companies. This paper proposes a cross-media collaborative filtering neural network model based on Deep FM for fast video click-through rate estimation. We use an RNN structure to process users' historical behaviors and data augmentation to process the training data. This paper proposes a short video click-through rate prediction model (MMIE) based on multimodal features and interest evolution. By analyzing the business scenarios in the fast video domain, this paper improves the structural unit of GRU by directly extracting short video multimodal features as video content representation and using attention mechanism in the processing of user behavior sequence features so that it can learn user interest evolution process with focus and improve the accuracy of click-through rate prediction. Experiments are conducted on the MMIE model, thus demonstrating the feasibility and effectiveness of the proposed model at the data level. The experimental results show that the MMIE model presented in this paper works best. In addition, many experiments are conducted on the way different features are combined, and the experiments show that the more elements are fused, the higher the accuracy rate the model can achieve.

## Figures and Tables

**Figure 1:** Flowchart of extensive data collection, processing, and storage of transmedia technology.

**Figure 2:** Collaborative filtering model of convolutional neural network with outer vector product.

**Figure 3:** Network structure of the click-through rate prediction model.

**Figure 4:** Comparison of disambiguation effects of different classification models with separate feature extraction.

**Figure 5:** NCF performance on Movie Lens-100k dataset.

**Figure 6:** Experimental results of MMIE and SDIN in different sequence length comparison.

**Figure 7:** Comparison of test results of different components.

**Table 1:** Audio feature extraction results.

Function number	Function name	Description
1	Chromaticity deviation	Standard deviation of 12 chromaticity coefficients
2	Chromaticity vector	The 12 elements of spectral energy represent the 12 isothermal pitch classes (semitone spacing) of Western music
3	Mel's inverse spectral coefficient	Mel frequency cepstrum coefficients forming the cepstrum representation, where the frequency bands are not linear but have to be distributed according to the Mel scale
4	Spectral roll-off point	Below this frequency, 90% of the spectrum's amplitude distribution is concentrated
5	Spectral flux	The squared difference between the normalized amplitudes of the spectra of two consecutive frames
6	Spectral entropy	The entropy of the normalized spectral energy of a set of subframes
7	Spectral extension	The second central moment of the spectrum
8	Spectral center of mass	The center of gravity of the spectrum
9	Energy entropy	The entropy of the normalized energy of a subframe, which can be interpreted as a measure of the mutation
10	Energy	The sum of squares of the signal values normalized by the corresponding frame length
11	Trans-zero rate	The rate of sign change of the signal during a given frame duration

## Data Availability

The data used to support the findings of this study are available from the corresponding author upon request.
